# Research on Real-Time Face Key Point Detection Algorithm Based on Attention Mechanism

**DOI:** 10.1155/2022/6205108

**Published:** 2022-01-05

**Authors:** Jiangjin Gao, Tao Yang

**Affiliations:** ^1^Information Technology Center, Chengdu Sport University, Chengdu 610041, China; ^2^Education and Information Technology Center, China West Normal University, Nanchong 637002, China

## Abstract

The existing face detection methods were affected by the network model structure used. Most of the face recognition methods had low recognition rate of face key point features due to many parameters and large amount of calculation. In order to improve the recognition accuracy and detection speed of face key points, a real-time face key point detection algorithm based on attention mechanism was proposed in this paper. Due to the multiscale characteristics of face key point features, the deep convolution network model was adopted, the attention module was added to the VGG network structure, the feature enhancement module and feature fusion module were combined to improve the shallow feature representation ability of VGG, and the cascade attention mechanism was used to improve the deep feature representation ability. Experiments showed that the proposed algorithm not only can effectively realize face key point recognition but also has better recognition accuracy and detection speed than other similar methods. This method can provide some theoretical basis and technical support for face detection in complex environment.

## 1. Introduction

Artificial intelligence has made great progress in bridging the gap between human and machine capabilities [1–3]. Face detection plays an important role in the field of artificial intelligence. Face key point detection is an important part of face detection. Face key point detection is defined as the detection and location of some feature points of the face [4, 5]. The commonly used key points are the corner of the eye, tip of the nose, corner of the nostril, corner of the mouth, eyebrow arc, earlobe, bridge of the nose, chin, etc. This is an important intermediate step in many subsequent facial processing operations, from biometrics to the understanding of mental state. Facial key point localization plays an important role. Typical applications are facial expression analysis, facial animation, 3D face reconstruction or registration, feature-based face recognition or verification, face tracking, and head pose understanding. The subsequent applications of face key points may be the anonymization of face identity in digital photos, image editing software tailored for face, lip reading, sign language interpretation, etc. Traditional methods (such as the first active shape model, improved model, active appearance model, further improved model, local constraint model, and more variants) try to obtain descriptors that can represent local features, so as to locate facial contour using heuristic rules [6–8]. Inspired by the previous coarse to fine regression model, cascade regression model was very popular in the first few years when deep learning began to prevail in computer vision. CRM abandons the classical machine learning algorithm, uses convolutional neural network, and gradually (even locally) refines the coordinates of key points, which proves that it is superior to the traditional methods. One of them is still multitask convolutional neural network, which is welcomed by many developers. However, under the influence of numerous human factors, when facing the unconstrained face images in the field (such as posture, occlusion, expression, lighting, makeup, blur, etc.), they are still far from a robust and accurate face key point location model [9, 10].

In recent years, face key point detection mainly focuses on two mainstream methods, namely, coordinate regression, heat map regression, and various model design. The coordinate regression model attempts to construct a mapping between the input face image domain and the coordinate domain, which is a naive and explicit way of end-to-end learning [11–13]. The multitask constrained depth convolution network believes that learning facial attributes can promote the positioning of key points, because these attributes (such as wearing glasses, smile, and head posture) can indicate the distribution of landmarks. The heat map regression model based on full convolution network outputs the heat map of each landmark and tries to maintain the structural information in the whole network. Therefore, to some extent, its most advanced performance is better than the coordinate regression model. The multiview hourglass module is one of these heat map regression models, which can continuously realize face detection and face alignment and use the stacked hourglass model to predict the heat map of key points [14, 15]. Face boundary information can recognize the geometric structure of human face. Therefore, whether it is used for attention mechanism or for generating boundary coordinate heat map, the network with a priori knowledge can be injected into the network.

According to the existing research, the main problems of face key point detection in the image have been basically solved. Under general conditions, the positioning accuracy of key points exceeds the human level, and it can show good robustness to occlusion, illumination, and other noises. However, for some extreme fuzzy and large angle facial images, they still cannot reflect good generalization ability, and the accuracy of key point location is far lower than that of human vision. Therefore, a real-time face key point detection algorithm based on attention mechanism is proposed in this paper. This paper studies the problems existing in the real-time detection of face key points, combines the attention mechanism with real-time detection, improves the ability of image feature extraction, and improves the stability and accuracy of the algorithm.

## 2. Related Works

### 2.1. Face Key Point Detection

The early face key point detection algorithms used parametric shape model method. The most classical traditional algorithms are active shape model algorithm and active appearance model algorithm. The first proposed active shape model algorithm abstracts the target object through the shape model [16, 17]. It is an algorithm based on the point distribution model. In the active shape model, the geometry of the target with similar shape can be expressed as a vector through the coordinate series of some key points, such as human face and hand. The active shape model algorithm needs to label the training data set manually, then get the shape model through training, and then use the matching of key points to complete the matching of specified targets. The active shape model algorithm is mainly divided into two stages: the first stage is training shape model: collecting training data; manually marking the key points on the face. The coordinates of key points in the training sample data are represented by shape vectors. The shape is processed by normalization and alignment. Principal component analysis was used to deal with the aligned shape features. In order to find a new location for each key point in each iterative search, local features are established for each key point. In order to deal with the change of illumination, the gradient feature is generally used as the local feature. The second stage is search: first calculate the position of eyes and mouth, carry out basic rotation change and scale change, and carry out preliminary face alignment. Then, in order to get the initial shape, search near the aligned points and match each local key point [18, 19]. The search matching process often uses Markov distance as an index. Then the shape model is used to modify the matching results. The above process is iterated until convergence. The active appearance model improves the active shape model by adding not only shape constraints, but also the texture features of the whole face region. Similar to active shape model, active appearance model is also divided into two stages: model establishment and model matching. In the modeling stage, in addition to the shape model of the training samples, the active appearance model also establishes the texture model and then combines the two models [20, 21]. The advantages of active shape model and active appearance model algorithm are clear architecture, simple model, strong constraints on contour shape, and being easy to understand. However, the disadvantage is that the location method of near exhaustive search key points limits its computational efficiency to some extent.

### 2.2. Attention Mechanism

Attention mechanism is similar to human vision. When objects appear, more attention will be paid to key information and useless information will be suppressed at the same time. In recent years, the relationship between computer vision tasks and attention mechanism has become increasingly close, such as residual network with attention mechanism for Alzheimer's disease (AD) recognition and classification [22]. A network with attention mechanism is used to detect bridges in synthetic aperture radar (SAR) images [23]. According to the different regions of attention, the attention mechanism can be divided into channel domain, spatial domain, and mixed domain. Squeeze and Exception Network (SENet) is a typical channel domain attention mechanism [24]. Through autonomous learning of each channel, it can identify the importance of each channel and actively enhance the weight of important channels. However, the dimensionality reduction operation contained in SENet will affect the channel correlation prediction, and the correlation capture of all channels will also reduce the efficiency of the network. The Spatial Transformer Networks proposed by Jaderberg et al. is a typical spatial domain attention mechanism, which can convert and save the spatial information in the image to another space [25, 26]. Revolutionary block attention module (CBAM) is a common hybrid domain attention mechanism [27]. By connecting the spatial domain and channel domain in series, the network performance can be improved more effectively.

Attention mechanism makes neural network pay more attention to the detailed information related to features, which can speed up the information processing time, improve the efficiency of computer processing information to a certain extent, and finally improve the expression ability of features. This paper selects the SENet attention mechanism, which learns the relationship between channels, then processes the feature map obtained by convolution, finally obtains a vector with the same dimension as the number of channels, and adds this vector to the corresponding channels as a weight number.

## 3. Proposed Method

### 3.1. Convolutional Neural Network

As one of the representative algorithms of deep learning, convolutional neural network imitates the visual mechanism of biology and has strong representational learning ability. A CNN is mainly composed of five structures: input layer, convolution layer, pooling layer, activation function, and full connection layer [28, 29]. Each layer has multiple feature maps, each feature map extracts an input feature through a convolution filter, and each layer except full connection is only connected to some nodes of its upper layer. In more complex networks, the structure of inception and residual block may appear in the network. For different research fields and directions, different dimensions of data need to be input into convolutional neural network. In the field of computer vision, the input of target detection is generally the three-dimensional pixel matrix of the image. For classification tasks, each node in the output layer usually represents the credibility of different categories.

The function of convolution layer is to extract the features of input data. The low-level convolution layer can only extract some features with low abstraction. With the increase of network depth, the extracted features will be more complex. Step *s* and filling size *p* are two important parameters in convolution layer. For the characteristic diagram with input size *w* × *h*, the output size is *w*′ × *h*′, and the calculation is shown in formulas (1) and (2):

(1) $$\begin{array}{c} w^{\prime }=\frac{2p+w-k}{s}+1, \end{array}$$

(2) $$\begin{array}{c} h^{\prime }=\frac{2p+h-k}{s}+1, \end{array}$$

where *k* is the size of convolution kernel, *s* is the step size, and *p* is the filling size.

In multilayer neural networks, the output of the previous layer is usually transformed by the activation function and then input to the next layer. Because the data in real life is often not linear, the activation function is usually a nonlinear function, which can effectively enhance the expression ability of the network and help to express complex features. Its expression form is shown in the following formula:

(3) $$\begin{array}{c} B_{x,y,z}^{m}=f\left(N_{x,y,z}^{m}\right), \end{array}$$

where *f* is the activation function, *z* is the convolution kernel, (*x*, *y*) is the pixel of the corresponding feature map, *N*^*m*^ is the convolution input of layer *m*, and *B*^*m*^ is the output of layer *m* convolution after activation function.

The pool layer is usually behind the convolution layer. Through downsampling, some unimportant information in the feature map is removed, to further reduce the number of parameters, reduce the size of the model, improve the calculation speed, and improve the robustness of the extracted features. The formula for calculating the size of convolution layer is also applicable to pool layer.

The full connection layer is located at the end of the convolution neural network. Its function is to classify the output obtained by nonlinear combination of the extracted features. Convolution extracts local features, while full connection combines all local features by weight. Generally speaking, the convolutional neural network will be followed by three full connection layers. In order to prevent overfitting during training, dropout is often added to the whole connection layer, and the activation value of some neurons in the whole connection layer is randomly set to 0.

### 3.2. Attention Module

Attention mechanism comes from the study of human vision. Human beings always selectively pay attention to some information and ignore other information. Therefore, the introduction of attention mechanism in deep learning is to help the network pay attention to some important global information and then combine it with local information. Attention mechanism [30] was proposed by Google in 2017 and began to be used in machine translation. Later, it was used in recommendation system [31, 32], character recognition [33, 34], semantic segmentation, natural language processing, and other aspects and achieved good results.

Hu j et al. proposed channel attention in SENet [35], by using two compressed full connection layers to learn the channel weight and then multiplying it with the original feature map for feature recalibration; the importance of each feature channel is automatically obtained through learning, so as to filter out unimportant features. Specifically, SENet learns the weight by reducing the loss value, so as to increase the weight of effective feature map and reduce the weight of invalid or small feature map, so as to improve the detection effect. The network structure of SENet is shown in Figure 1.

The whole module is divided into two operations: Squeeze and Excitation. The Squeeze operation converts the characteristic graph of *h* × *w* × *n* into the output of 1 × 1 × *n* by using global average pooling, obtains the global receptive field, and matches the dimension of the output with the input. The calculation is shown in formulas (4) and (5):

(4) $$\begin{array}{c} N_{n}=F_{c}\left(g_{n}\right), \end{array}$$

(5) $$\begin{array}{c} F_{c}\left(g_{n}\right)=\frac{1}{h\times w}\sum_{x=1}^{h}\sum_{y=1}^{w}g_{n}\left(x,y\right), \end{array}$$

where *n* represents the number of channels, *h* and *w* represent height and width, respectively, and *g*_*n*_ is the *n*-th two-dimensional matrix in *g*.

The Excitation operation first performs full connection and then scaling to reduce the number of channels, thus reducing the amount of calculation. Make another full connection back to the original number of channels, which increases the nonlinear ability of the network and can better fit the complex relationship in the characteristics. The calculation is shown in formulas (6)–(8):

(6) $$\begin{array}{c} w_{s}=F_{d}\left(w_{z}\right), \end{array}$$

(7) $$\begin{array}{c} F_{d}\left(w_{z}\right)=\text{sig}\left(q\left(w_{z}\right)\right), \end{array}$$

(8) $$\begin{array}{c} \text{sig}\left(q\left(w_{z}\right)\right)=\text{sig}\left(w_{1}\rho \left(w_{2}\right)\right), \end{array}$$

where *w*_*s*_ is the learned characteristic graph weight, and *w*_1_ and *w*_2_ are the fully connected weight parameters. sig represents sigmoid activation function and *ρ* represents ReLU activation function.

After the operation of Squeeze and Excitation, the weight *w*_*s*_ of the obtained feature map is multiplied by the original feature map pixel by pixel; that is, the global attention information is added to the feature map to complete the feature recalibration on the number of channels. The calculation is shown in the following formula:

(9) $$\begin{array}{c} B=F_{e}\left(g_{n},w_{sn}\right). \end{array}$$

SENet not only is simple to implement, but also has strong universality. It can be inserted into different classification or detection networks and has achieved good results. However, compared with the fact that SENet only focuses on channel attention, Woo et al. proposed the Convolutional Block Attention Module (CBAM) [27], which combines the spatial attention module and channel attention module to achieve better results. The CBAM network structure is shown in Figure 2.

Firstly, the spatial attention module pools the feature map with the size of *h* × *w* × *n* based on the channel to obtain the feature map with the size of *H* × *W* × 1. Secondly, concatenate the two feature maps and then perform a convolution operation to reduce the dimension to one channel. Finally, the spatial attention feature map is generated by sigmoid activation function.

The channel attention module pools the feature map with the size of *h* × *w* × *n* based on height and width to obtain the feature map with the size of 1 × 1 × *n*, after adding the two feature maps pixel by pixel and then generate the channel attention feature map through the sigmoid activation function. CBAM module can be embedded into most target detection models, increase the feature extraction ability of the network, and significantly increase the detection accuracy without increasing the amount of calculation.

### 3.3. Overall Network Construction

Due to the diversity of face key feature points, multiscale feature map is used for prediction, and attention mechanism is introduced into the network. This paper adopts the deep convolution network model [36, 37]. The VGG network structure is shown in Figure 3. The number of network layers often uses 16 layers, that is, VGG16 to complete the experiment. The 16 layers contain 13 convolution layers and the last three fully connected layers, by stacking multiple 3 × 3 convolution kernels instead of a large-size convolution kernel and using multiple continuous convolution layers. The small-size convolution kernel must have small receptive field. The purpose of using large-size convolution kernel instead is to increase the receptive field and reduce the required training parameters. By stacking two 3 × 3 convolution cores to replace one 5 × 5 convolution core and docking three 3 × 3 convolution cores to replace one 7 × 7 convolution core, the receptive field with the same size as the large convolution core can be achieved by stacking small-size convolution cores. You can see the network structure when the input picture size is 224 × 224 and the number of channels is 3.

The network structure of VGG model and the dimensions and levels corresponding to the characteristic diagram of each layer are shown in Table 1.

Because the traditional face detection method will use a candidate box, which is generated through a sliding window, there will be a lot of redundancy when extracting the target candidate region. Therefore, NMS (nonmaximum suppression) is used to eliminate redundant frames when detecting face key features. As shown in Figure 4, due to the sliding window, we may get a lot of rectangular boxes, including the face area we need. Obviously, these rectangular boxes represent the same goal, and NMS algorithm can remove these redundant boxes.

When using deep learning target detection algorithm, NMS algorithm will also be used to remove some redundant candidate boxes. Firstly, when using the classifier for classification, we will get a probability value, which is expressed as the idea that the current detection box is the probability value of the detection target we need, and sort it to get the corresponding score. Then, after sorting all the detection boxes with the score value, select the detection box with the largest score, and delete the boxes whose IOU area is greater than some threshold; that is, the overlap rate is high.

### 3.4. Multiscale Feature Fusion

Compared with general target detection backbone networks, such as VGG network, it is characterized by multilevel feature extraction, which is called feature graph. CNN can be considered as a process of extracting high-level semantic features [38, 39]. When face recognition is carried out, the bottom features only represent some facial contour features, such as size and shape, but the high-level features are often more detailed features, such as eyes, mouth, and other facial features. When it comes to recognition, they represent a feature of the whole face. For VGG networks, the deeper the features are, the more abstract the representation is, the more favorable the classification task is, and the stronger the semantic information is, but at the same time, the lower the resolution is, which is not conducive to the detection of small targets. Generally speaking, the low-level feature has high resolution but weak semantic information, and the high-level feature has strong semantic information and low resolution, which is not conducive to detection. Although the semantic information of the underlying features is weak, the amount of information is large enough. However, at the high level, due to many convolution operations, the feature dimension becomes smaller and smaller, which may lose a large part of the information of small targets, which limits the detection accuracy of small targets. The key points of the face are visualized in each layer, as shown in Figure 5, which is the visualization results from layer 1 to layer 16.

The functions of each layer can be understood from the characteristic diagrams visualized from different layers. In this paper, the feature fusion method is used to solve this problem. The basic method is to transfer the information of the previous layer network to the next layer network, so that the features of the previous layer can still be supplemented after convolution operation, reduce the loss of feature information, and make the small target features more complete. It has both location information and strong semantic information. When the high-level features are removed and upsampled, the feature map becomes larger and the semantic information becomes stronger. The low feature horizontal links are added to the corresponding feature map to obtain a top-down multiple feature fusion network.

### 3.5. Face Key Points Training and Recognition

The above network structure is mainly used to complete face classification, key feature detection, and frame detection. Therefore, it is necessary to extract the key points of the face and calibrate the position [40–42]. Using the selected samples in the database, the network is trained and the key points are obtained. Three training tasks are completed through the network structure to determine whether it is a face, detect the position of the face, and locate the key points of the face. Finally, it is connected and output through the full link layer, and the network parameters are optimized and updated through the loss function.

In order to detect whether it is a face and its key features, the final output layer uses the cross direct function to realize the classification of face key feature detection. The classification error values after training are as follows:

(10) $$\begin{array}{c} L_{a}=-\left({\hat{x}}_{a}\log\left(\frac{1}{1+e^{-\alpha_{0}}}\right)\right)+\left(1-{\hat{x}}_{a}\right)\left(1-\log\left(\frac{1}{1+e^{-\alpha_{1}}}\right)\right), \end{array}$$

where ${\hat{x}}_{a}$ denotes the real label of its background, *α*_0_ and *α*_1_ are the correlation coefficient, and its value is determined by experiment.

When detecting the position of face key points, the predicted relative position of face key points can be obtained through the network. The Euclidean calculation is carried out by using the predicted position of the face and the calibrated actual position, to calculate the loss value of the position frame, as shown in formula (11), and the value is minimized by iteratively updating the parameters:

(11) $$\begin{array}{c} L_{b}={\left\|{\hat{x}}_{b}-x_{b}\right\|}_{2}. \end{array}$$

For face key point location, the five key feature points of the face can be predicted through the network, and the L2 norm is calculated with the calibrated feature positions, to calculate the loss value of face key points, as shown in the following formula:

(12) $$\begin{array}{c} L_{c}={\left\|{\hat{x}}_{c}-x_{c}\right\|}_{2}. \end{array}$$

Finally, the final loss function is obtained by calculating the values and corresponding weights through formulas (10) and (12), which can be expressed as follows:

(13) $$\begin{array}{c} L\left(x_{m}\right)=\sum_{n\in \left\{a,b,c\right\}}\eta_{m}\lambda_{n}L_{m}^{n}, \end{array}$$

where *η*_*m*_ and *λ*_*n*_ denote the weighting coefficient, and its value is determined by experiment.

Using the iterative training results of the network model, the false alarm samples generated in each stage are put into the next batch of training samples to ensure more accurate network identification. The face detection algorithm under the above deep learning framework is used to add the face recognition function [43]. The face recognition adopts the SVM algorithm for 1-to-1 comparison, as shown in Figure 6, which is the flowchart of SVM face training and recognition.

## 4. Experiment and Analysis

### 4.1. Data Set Selection and Processing

We select 300W-LP [44], WFLW [45], and AFLW2000-3D [46] as the generator, that is, the training set of image face key point detection. At the same time, they are used as a test data set to evaluate the accuracy of face key location points.

300w-LP data set generates large angle side face images with a full range of −90° to 90° by 3D rotation transformation and rerendering of the existing integrated data set 300W. The whole data set contains 61225 images, the original image size is 450 × 450, and it contains 68-point type key point annotation data of 2D and 3D.

WFLW data set contains 10000 faces (7500 photos for training and 2500 photos for testing) and 98 completely manually labeled keys. In addition to key point annotation, the new data set also contains rich attribute annotations, namely, occlusion, pose, makeup, lighting, blur, and expression, which can comprehensively analyze the existing algorithms.

AFLW2000-3D data set contains 2000 face images with coordinate annotation of 68 3D face key points. The annotation is automatically generated by the 3D reconstruction algorithm of the face, and the variation range of the face side angle is (−90°, 90°). Due to the defects of the automatic annotation generation method, the annotation of some images is not very accurate, but the NME index on the data set is still the most widely used 3D face key point positioning accuracy evaluation method at present.

300W-LP, WFLW, and AFLW2000-3D data sets are used for experiments, and the data sets are shown in Table 2.

The video contained in 300W-LP, WFLW, and AFLW2000-3D data sets is read by Opencv and saved for 30 frames. After the obtained image frames are aligned and cut by Mtcnn face, the image frame size is normalized to 125 × 125 RGB image.

### 4.2. Results

In practical application, the preset task of face frame detection is required before face key point detection. The input of stacked hourglass network is the truncated face image. In the ideal case of frame detection, the face is centered relative to the image frame, and the face size ratio is fixed. Therefore, the key point detection network does not need to show strong generalization ability to the changes of offset and scaling in a wide range. When processing 300w-LP image training data, first determine the face frame according to the key point coordinates given by it, and then enlarge it to a certain proportion to ensure that all face pixel information is selected.

For the image with the given key point coordinate marked as {*X*_*i*_=(*x*_*i*_, *y*_*i*_),  *i*=1,2,…, 68}, the center coordinate (*x*_*n*_, *y*_*n*_) and frame variable length *m* of the face box we finally cut out have the following calculation formulas:

(14) $$\begin{array}{c} x_{\max}=\max\left(x_{i}\right),\\ x_{\min}=\min\left(x_{i}\right),\\ y_{\max}=\max\left(y_{i}\right),\\ y_{\min}=\min\left(y_{i}\right),\\ x_{n}=\left\lfloor \frac{x_{\max}+x_{\min}}{2}\right\rfloor ,\\ y_{n}=\left\lfloor \frac{y_{\max}+y_{\min}}{2}\right\rfloor ,\\ m=\left\lceil \frac{3\left(\max\left(x_{\max}-x_{\min},y_{\max}-y_{\min}\right)\right)}{2}\right\rceil . \end{array}$$

After intercepting the face box, we call the standard library function to scale and sample it to the standard input size *w* × *h* of the network, where we all select 256. This step can be regarded as the pretask of simulating face frame detection by using the labeled coordinate information to ensure that the input of key point detection network has good consistency.

In order to make VGG and other neural network models have better generalization ability, this paper uses the data enhancement method to transform the input data in order to generate more training data with a wider range of hidden parameters. Due to the symmetry of face, the training data can be doubled directly by turning the image left and right, and the problem of uneven distribution of left and right face data can be overcome. Although the input images are all centered images with fixed proportion after preprocessing, in order to enable the model to deal with certain pretask errors and deal with the input of nonstandard interception in video continuous frames, it is still necessary to enhance the translation and scaling in a small range, and the selected translation random quantity is [−0.3 m, 0.3 m], and the random scaling is [0.8, 1.6]. The 2D rotation of [−45°, 45°] relative to the face center further enhances the face pose. Translation, scaling, and rotation can be combined into an affine transformation, which acts on the pixel index and key coordinates at the same time.

Table 3 shows the NME values of the generator on the test data set trained by the method in this paper, including the pretrained model and the model after stability enhancement. NME references of some benchmark algorithms are also given in Table 3.

In addition, this paper uses data sets for training and testing, respectively. In quantitative analysis, the experiment uses accuracy rate (AR) and misjudgment rate (MR) as the evaluation indexes of the algorithm. When quantitatively analyzing the real-time performance of face detection and recognition, this paper verifies the performance of the algorithm by the time required for the system to process a frame of image and CPU occupancy. Comparison results of accuracy of different algorithms on each data set are shown in Table 4.

The results show that the accuracy is improved. The experimental results of different algorithms on various data sets show that this method is superior to other algorithms in various indexes.

In order to show that the pretraining designed in this paper is indeed helpful to make the model obtain better generalization ability, a video on the Internet is selected, and some difficult frames in which it is difficult to locate face key points are extracted for comparative test. The results are shown in Figure 7.

It can be seen that the proposed model cannot guarantee the positioning accuracy but still maintains a clear face structure when dealing with such large angle occlusion and motion blur. However, models without confrontation training, such as fan, do not have such generalization ability due to the lack of diversity of image training set itself.

### 4.3. Discussion

As a basic task in the field of computer vision, face key point detection has always been the research focus of scholars [52]. The existing face detection algorithms based on anchor box have some disadvantages. Firstly, too many anchor boxes need to be preset, which consumes computing resources and time. Secondly, the shape of the anchor box depends on the preset rectangle, which will make the detection effect of face key points worse. Finally, many superparameters will increase the difficulty of training the algorithm. Therefore, face key point detection based on nonanchor box has become a research hotspot of scholars in recent years [53]. The benchmark model algorithm VGG in this paper is one of many nonanchor frame target detection algorithms, and the benchmark model algorithm also has some problems: (1) It is more affected by background texture information because it depends on key points. (2) Because more attention is paid to the corner information and the center information is not fully utilized, the final inspection is missed. This paper improves the algorithm for the above problems and solves the above problems to a certain extent. Because the benchmark algorithm VGG is based on three key points: the upper left corner, the lower right corner, and the center point, the complex background texture information in the image will have an adverse impact on the key point detection [54]. To solve this problem, this paper proposes to add the expectation maximization attention mechanism to the benchmark algorithm to reconstruct the extracted feature map, weaken the background texture information, and strengthen the foreground information. Experiments show that the accuracy of this method is higher than that of the benchmark algorithm.

## 5. Conclusion

Starting from the computer vision task of face key point recognition, the key point detection of existing high accuracy models in real-time application scenarios may be ambiguous or incomplete, resulting in feature loss. Therefore, a real-time face key point detection algorithm based on attention mechanism is proposed to solve the problem of multiscale face feature detection. In the standard VGG framework, for the multiscale face key point features, the feature enhancement module and feature fusion module are used to improve the shallow feature representation ability in VGG. At the same time, a cascade attention mechanism is adopted to highlight the target of the spatial region on the given feature map. By improving the deep feature representation ability, the network is more conducive to the recognition of face key point features. For directly related visual tasks such as real-time detection of human key points and real-time detection of object key points, similar methods are considered to be improved. The more difficult step is to obtain a parametric 3D object model like 3DMM. Considering that face key point detection is only a subclass that is easy to implement in the face comparison task and the comparison of more fine-grained face models, such as the accuracy of face 3D reconstruction, is still not ideal, we still have a long way to go in order to make machine vision have the understanding ability close to human vision in face images [55, 56].

## Figures and Tables

**Figure 1:** The network structure of SENet.

**Figure 2:** The network structure of CBAM.

**Figure 3:** The network structure of VGG.

**Figure 4:** Schematic diagram of nonmaximum suppression algorithm.

**Figure 5:** Schematic diagram of feature visualization results of different layers.

**Figure 6:** Flowchart of SVM face key points training and recognition.

**Figure 7:** Flowchart of face key points extraction and recognition.

**Table 1:** Characteristic diagram parameters of VGG network structure.

Number of layers	Characteristic diagram	Number of layers	Characteristic diagram
First layer	224 × 224 × 64	Ninth layer	28 × 28 × 512
Second layer	224 × 224 × 64	Tenth layer	28 × 28 × 512
Maximum pool layer	112 × 112 × 128	Maximum pool layer	14 × 14 × 512
Third layer	112 × 112 × 128	Eleventh layer	14 × 14 × 512
Fourth layer	112 × 112 × 128	Twelfth layer	14 × 14 × 512
Maximum pool layer	56 × 56 × 256	Thirteenth layer	14 × 14 × 512
Fifth layer	56 × 56 × 256	Maximum pool layer	7 × 7 × 512
Sixth layer	56 × 56 × 256	Fourteenth layer	1 × 1 × 4096
Seventh layer	56 × 56 × 256	Fifteenth layer	1 × 1 × 4096
Maximum pool layer	28 × 28 × 512	Sixteenth layer	1 × 1 × 1000
Eighth layer	28 × 28 × 512	Output	

**Table 2:** The training set and testing set of each data set required for the experiment.

Data set	Number of samples		
	Training set	Testing set	Total
300W-LP	3500	1300	4800
WFLW	2400	1200	3600
AFLW2000-3D	2800	1300	4100

**Table 3:** Performance comparison results of different algorithms on each data set.

Algorithm	Angle range				Mean
	[0,20)	[20,40)	[40,60)	[60,80)	
SqueezeNet [47]	2.72	3.46	4.74	6.74	4.42
Xception [48]	2.53	3.68	4.51	5.92	4.16
LBP [49]	3.75	4.23	5.35	7.49	5.21
ShuffleNetV2 [50]	2.46	3.84	4.73	6.43	4.37
MobileNetV2 [51]	3.62	4.45	5.22	7.37	5.17
This method	2.24	3.13	4.34	5.28	3.75

**Table 4:** Comparison results of accuracy of different algorithms on each data set.

Algorithm	300W-LP		WFLW		AFLW2000-3D	
	AR (%)	MR (%)	AR (%)	MR (%)	AR (%)	MR (%)
SqueezeNet [47]	95.61	4.39	96.48	3.52	96.83	3.17
Xception [48]	93.45	6.55	95.23	4.77	95.37	4.63
LBP [49]	95.68	4.32	96.37	3.63	96.51	3.49
ShuffleNetV2 [50]	94.52	5.48	95.42	4.58	94.37	5.63
MobileNetV2 [51]	97.28	2.72	97.48	2.52	94.59	5.41
This method	98.27	1.73	98.36	1.64	97.48	2.52

## Data Availability

The labeled data set used to support the findings of this study is available from the corresponding author upon request.
